The article "Poricoic Acid A Inhibits the NF-κB/MAPK Pathway to Alleviate Renal Fibrosis in Rats with Cardiorenal Syndrome" was retracted in 2023. Reasons: signs of a paper mill; suspected computer-generated content; unreliable results or conclusions; concerns about the data.

# Poricoic Acid A Inhibits the NF-*κ*B/MAPK Pathway to Alleviate Renal Fibrosis in Rats with Cardiorenal Syndrome

**DOI:** 10.1155/2022/8644353

**Published:** 2022-06-15

**Authors:** Wenzhong Chen, Zhiwen Fan, Canhui Huang, Junying Liu

**Affiliations:** ^1^Department of Cardiovascular Medicine, Guangzhou First People's Hospital, School of Medicine, South China University of Technology, Guangzhou, Guangdong 510180, China; ^2^Department of Cardiology, The PLA 74th Group Army Hospital, Guangzhou, Guangdong 510300, China; ^3^Department of Endocrinology, The First Affiliated Hospital of Shenzhen University, Health Science Center, Shenzhen Second People's Hospital, Shenzhen, Guangdong 518000, China

## Abstract

**Objective:**

To explore the potential and mechanism of action of poricoic acid A (PAA) in treatment of cardiorenal injury and fibrosis due to cardiorenal syndrome (CRS).

**Materials and Methods:**

A CRS rat model was established by transabdominal subtotal nephrectomy (STNx). The experimental group was treated by gavage of PAA (10 mg/kg/day). After 8 weeks of treatment, echocardiography was utilized for detecting heart-related indexes in rats. HE and Masson staining were conducted to detect the degree of pathological damage and fibrosis in rat kidney tissue, respectively. In addition, serum blood urea nitrogen (BUN), serum creatinine (SCr), and 24-hour urine protein were measured biochemically. Also, the levels of inflammatory factors (IL-1*β*, IL-6, and IL-10) in rat kidneys were measured using ELISA. Western blot was used to examine the expression of NF-*κ*B/MAPK pathway-related proteins.

**Results:**

In this study, a CRS rat model was successfully established by STNx surgery. PAA treatment could significantly alleviate the damage of heart and kidney function in CRS rats and reduce the pathological damage of kidney tissue and renal fibrosis. Meanwhile, PAA could also inhibit the renal inflammatory response through downregulating IL-1*β* and IL-6 levels in the kidney tissue and upregulating IL-10 level. Further mechanism exploration showed that the NF-*κ*B/MAPK signaling pathway was significantly activated in CRS rats, while PAA treatment could markedly inhibit the NF-*κ*B/MAPK signaling pathway activity in CRS rats.

**Conclusion:**

PAA can obviously improve the pathological damage and fibrosis of renal tissue in CRS rats and maintain the function of the heart and kidney. The above functions of PAA may be achieved by inhibiting the NF-*κ*B/MAPK signaling pathway activity. Briefly speaking, PAA can serve as a potential drug for CRS treatment.

## 1. Introduction

Cardiorenal syndrome (CRS) commonly refers to the heart and kidney damage caused by a series of feedback mechanisms due to collective dysfunction of the heart and kidneys. CRS was first mentioned at the working group of the National Heart, Lung, and Blood Institute in 2004, and the interaction between heart and kidneys was also assessed in this conference [1, 2]. Studies have shown that even mild renal impairment is associated with a significant increase in cardiovascular disease-related morbidity and mortality [3]. Following different criteria, the Acute Dialysis Quality Group categorized CRS at a consensus meeting. Specifically, CRS was divided into cardiorenal and renocardiac syndromes according to the main activity of the disease process. While according to disease severity and order of organ involvement, CRS was classified into five subtypes (type 1–5 CRS). These 5 subtypes included all cardiorenal damage caused by systemic diseases [4]. As statistics showed, the global prevalence of chronic kidney disease (CKD) was approximately 323 million in 2015. Therefore, cardiovascular disease was the leading cause of death among CRS populations [5]. At present, there are different clinical treatment plans for different classifications of CRS patients, including surgery and diuretic-related drugs. However, current drug treatments are prone to drug resistance and poor prognosis [6]. Moreover, the underlying mechanisms of CRS remain unclear, so the options in the current treatment are limited. Considering the above dilemma, it is an urgent need to improve the treatment and prognosis of CRS by finding new therapeutic targets, developing more effective treatment methods, or finding effective new drugs.

The article "Poricoic Acid A Inhibits the NF-κB/MAPK Pathway to Alleviate Renal Fibrosis in Rats with Cardiorenal Syndrome" was retracted in 2023. Reasons: signs of a paper mill; suspected computer-generated content; unreliable results or conclusions; concerns about the data.

At present, a large number of natural products are applied for the treatment of diseases related to the heart, kidney, and liver [7]. *Poria cocos*, a well-known traditional medicinal fungus, grows around the roots of pine trees in Asia and North America [8]. Studies have revealed that *Poria cocos* extraction has a protective effect on renal fibrosis [9]. As the main active substance in *Poria cocos*, poricoic acid A (PAA) is a class of triterpenoids. Studies have observed that PAA has a strong diuretic effect and can be adopted to treat edema, kidney disease, dizziness, nausea, vomiting, etc. [10]. Studies have also revealed anticancer effects of PAA. For example, Ma et al. found that PAA could inhibit the proliferation, migration, and invasion of ovarian cancer cells SKOV3 and induce apoptosis and autophagy of cancer cells [11]. In addition, PAA plays an important role in a variety of kidney-related diseases. As found by Chen et al., PAA regulated nuclear factor-*κ*B (NF-*κ*B) and nuclear factor-erythroid-2-related factor 2 (Nrf2) pathways to reduce oxidative stress and inflammation, thereby improving renal fibrosis and podocyte injury in rats with renal ischemia-reperfusion injury (IRI) [12]. Meanwhile, Chen et al. also discovered that combination treatment of PAA and melatonin could affect the interaction of TGF-*β*/Smad and Wnt/*β*-catenin, thereby improving renal IRI and repairing hypoxia/reoxygenation or TGF-*β*1-induced HK-2 cell damage [13]. Furthermore, the effects of PAA have also been explored based on unilateral ureteral obstruction, 5/6 nephrectomy animal models, and TGF-*β*1-induced renal fibroblasts. Specifically, PAA, through AMPK activation and further Smad3 inhibition, inhibits accumulation and remodeling of abnormal extracellular matrix (ECM), promotes the inactivation of fibroblasts, and then improves renal function and inhibits renal fibrosis [14]. The above findings have suggested the therapeutic potential of PAA for renal damage and fibrosis. At present, there is no relevant research on the effect of PAA on central renal injury in CRS. Therefore, in this study, a CRS rat model was constructed by STNx surgery. Besides, the effects of PAA on cardiac and renal function, tissue damage, fibrosis, and inflammatory responses in CRS rats were explored *in vivo*. Also, the possible mechanism of action of PAA was further explored. The objectives of this study were to look for new drugs for the treatment of CRS and provide effective trial data support.

The article "Poricoic Acid A Inhibits the NF-κB/MAPK Pathway to Alleviate Renal Fibrosis in Rats with Cardiorenal Syndrome" was retracted in 2023. Reasons: signs of a paper mill; suspected computer-generated content; unreliable results or conclusions; concerns about the data.

## 2. Materials and Methods

### 2.1. Establishment and Treatment of the CRS Rat Model

The animal experiments described in this study were authorized by the experimental animal ethics committee of Guangdong Medical Experimental Center (2022–03). PAA was purchased from Nature Standard. Twenty-four adult SD rats (body weight: 180–220 g) were provided by Beijing Vital River Laboratory Animal Technology Co., Ltd. Then, the rats were randomly divided into 4 groups (Sham group, PAA group, CRS group, and CRS + PAA group), with 6 rats for each group. Transabdominal subtotal nephrectomy (STNx) was utilized for the establishment of CRS model rats, and the specific method was shown in the study of Cao et al. [15]. In the Sham group, sham surgery was performed in rats anesthetized by intraperitoneal (IP) injection of pentobarbital sodium (50 mg/kg), and the surgery steps were the same as STNx. However, the right renal artery, vein, and ureter were not ligated, the right kidney was not resected, and the left renal artery branch was not ligated. Then, the rats were gavaged with equal-volume distilled water. In the PAA group, sham surgery was performed followed the method of the Sham group and then 10 mg/kg/day of PAA was administered by gavage. In the CRS group, a CRS rat model was established by STNx surgery, and then, the rats were gavaged with an equal volume of distilled water. In the CRS + PAA group, a CRS rat model was established by STNx surgery and 10 mg/kg/day of PAA was gavaged for treatment. An 8-week experimental period was set for all groups. After the treatment, echocardiography was utilized for the examination of rats in each group. Then, the rats were euthanized. Finally, the heart tissue, tibia, kidney tissue, blood, and 24h urine of the rats in each group were collected for testing.

The article "Poricoic Acid A Inhibits the NF-κB/MAPK Pathway to Alleviate Renal Fibrosis in Rats with Cardiorenal Syndrome" was retracted in 2023. Reasons: signs of a paper mill; suspected computer-generated content; unreliable results or conclusions; concerns about the data.

### 2.2. Echocardiography

After the treatment, the limbs of the completely anesthetized rats in each group were fixed on the operating table. The rats lay on the left side of the table; then, after shaving chest hair, a small amount of couplant was applied. Small animal echocardiography was performed for the observation of left ventricular wall thickness and wall motion, as well as the measurement of left ventricular ejection fraction (LVEF), left ventricular end-diastolic volume (LVEDV), left ventricular end-systolic volume (LVESV), and left ventricular posterior wall thickness (LVPED) in rats of each group. Subsequently, we recorded the inner diameters of left ventricular end-systole and end-diastole, as well as the thicknesses of left ventricular posterior wall end-diastole and end-systole. The corresponding indexes were calculated as follows: LVEF = (LVEDV − LVESV)/LVEDV × 100%.

### 2.3. Heart Weight/Body Weight Ratio (HW/BW) and Left Ventricle/Tibia Length (LV/TL)

Heart weight/body weight ratio (HW/BW) and left ventricle/tibia length (LV/TL) were utilized to assess the degree of cardiac hypertrophy and left ventricular hypertrophy (LVH), respectively [16]. Precooled saline was injected into the left ventricle of euthanized rats until the heart was pale. Then, the heart was rapidly excised and flushed with normal saline (NS). Afterwards, the BW and HW of the rats were measured. Subsequently, the right ventricle tissue was removed along the interventricular septum. Then, the left ventricle weight (LVW) was checked and the tibia length (TL, cm) was measured. The HW/BW and LVW/TL of rats were calculated as follows:

(1) $$\begin{array}{c} \frac{HW}{BW}=\frac{HW}{BW\times 100\;\%};\frac{LVW}{TL}=\frac{LVW}{TL\times 100\;\%}. \end{array}$$

### 2.4. Biochemical Detection

The rats in each group were housed in metabolic cages (Sable Systems International, USA), respectively; 24 h urine was collected, and the total volume was calculated. Afterwards, 3 mL urine was taken out and centrifuged at 4 C and 3000 r/min for 10 min and then the supernatant was collected. After that, the peripheral blood of the rats in each group was collected through the tail vein. Then, the blood was centrifuged at 3000 r/min for 20 min and the upper serum was collected and separately placed into new centrifuge tubes for testing. A fully automatic biochemical analyzer (Olympus, Japan) was applied to check the urine protein (24-up) level in urine and the blood urea nitrogen (BUN) as well as the serum creatinine (SCr) level.

The article "Poricoic Acid A Inhibits the NF-κB/MAPK Pathway to Alleviate Renal Fibrosis in Rats with Cardiorenal Syndrome" was retracted in 2023. Reasons: signs of a paper mill; suspected computer-generated content; unreliable results or conclusions; concerns about the data.

### 2.5. Kidney Index

Kidney weight/body weight **(**KW/BW) was utilized to evaluate kidney function. Specifically, routine dissected operation was performed on the euthanatized rats to collect and mark kidney tissues. Then, the kidney tissues were weighed to calculate the kidney index.

### 2.6. HE Staining

The collected rat kidney tissues of each group were washed with phosphate-buffered saline (PBS) buffer, and the renal capsules were removed. Then, the tissues were fixed with 10% formalin and embedded with paraffin. Afterwards, the tissues were cut into sections with a thickness of 5 *μ*m. The sections were stained according to the instructions of the hematoxylin and eosin (HE) staining kit (Beyotime Biotechnology, China). To be specific, the sections were first stained with hematoxylin at 25°C for 5 min and differentiated with hydrochloric acid alcohol. Then, the sections were blued using 1% ammonia. After washing with distilled water, the sections were stained with eosin for 30 s, followed by alcohol dehydration and other steps. Finally, xylene-treated sections were mounted, then the kidney pathological changes were observed under a light microscope and photographed.

### 2.7. Masson Staining

Masson staining was applied to determine collagen deposition in the renal interstitium. Specifically, previously treated sections were collected for routine Masson staining according to the instructions of Masson's trichrome staining kit (Solarbio, China). Then, the pathological changes of kidney tissue and collagen fibers were observed and photographed under a light microscope. Blue collagen precipitation was regarded as a positive signal.

### 2.8. ELISA Detection

A total of 50 mg of kidney tissue were added to PBS buffer, fully homogenized in a tissue homogenizer, and centrifuged at 4 C, 12000 r/min for 30 min. After that, the supernatant was collected for testing. The level of interleukin (IL)-1*β*, IL-6, and IL-10 in the kidneys of rats in each group was determined according to the instructions of the corresponding ELISA detection kit (Nanjing Jiancheng, China).

### 2.9. Western Blot

The kidney tissues (50 mg) were added into radioimmunoprecipitation assay (RIPA) buffer (Beyotime Biotechnology, China) and homogenized at low temperature in a tissue homogenizer. Subsequently, the total protein was collected. The concentration of total proteins was determined according to the instructions of BCA protein assay kit (Thermo Fisher, USA). Subsequently, 10% sodium dodecyl sulphate-polyacrylamide gel electrophoresis (SDS-PAGE) was applied to separate 20 *µ*g of proteins in immunoblotting. After that, the proteins were electrotransferred onto a polyvinylidene fluoride (PVDF) membrane. Then, the membrane was blocked in 5% nonfat dry milk for 1–3 h. After washing, primary antibodies were added for incubation overnight at 4°C. Furthermore, the corresponding secondary antibodies were added for 1-h incubation overnight at 25°C after washing again. Finally, electrochemiluminescence (ECL) luminescence solution was dripped into the washed membranes for exposure in a protein imager, and then images were collected. In addition, GAPDH was used as an internal control and Image Lab^TM^ software was used for the analysis of the relative expression level of proteins.

The article "Poricoic Acid A Inhibits the NF-κB/MAPK Pathway to Alleviate Renal Fibrosis in Rats with Cardiorenal Syndrome" was retracted in 2023. Reasons: signs of a paper mill; suspected computer-generated content; unreliable results or conclusions; concerns about the data.

### 2.10. Statistical Analysis

All results in this paper were expressed as mean ± standard deviation (SD) and plotted by GraphPad Prism 9.0. SPSS 24.0 software was used to perform one-way analysis of variance for comparison between the multiple groups. *P* < 0.05 was considered as the criterion for judging the significance of differences.

## 3. Results

### 3.1. PAA Improves Cardiac Function Damage in Rats with Cardiorenal Syndrome (CRS)

To observe the effect of PAA on cardiac function in CRS rats, we first evaluated the effect of PAA on the cardiac function-related indices (LVEF, LVEDV, LVESV, and LVPED) of CRS rats using echocardiography. To be specific, compared with the Sham group, LVEF and LVEDV in the CRS group decreased significantly, while LVESV and LVPED increased notably. Besides, the ratios of HW/BW and LV/TL were markedly increased in the CRS group. The above suggested that the heart of the rat in the CRS group was hypertrophied, with impaired function, and the establishment of CRS model was successful. Additionally, no significant differences were observed in the above parameters between the Sham group and the PAA group, indicating that there were few effects of PAA treatment on the above parameters in rats with sham surgery. However, the CRS rats treated with PAA exhibited a remarkable decrease in the LVEF, LVEDV, LVESV, and LVPED. Also, the ratios of HW/BW and LV/TL were also obviously declined (Figure 1(a)–1(f)). All in all, PAA could notably improve cardiac hypertrophy and cardiac function damage in CRS rats.

### 3.2. PAA Alleviates Renal Function Damage in Rats with Cardiorenal Syndrome

Studies showed the association of renal injury with increased level of blood urea nitrogen (BUN) *in vivo*, serum creatinine (SCr), 24-hour urine protein (24-up), and elevated renal index KW/BW [17–19]. In order to assess the effect of PAA on renal damage in CRS rats, a fully automatic biochemical detector was used for the determination of the level of renal function-related indicators (BUN, SCr, and 24-up) of rats in each group. The outcome revealed that BUN, SCr, 24-up, and KW/BW were remarkably higher than those in the Sham group (*P* < 0.01),while the BUN, SCr, 24-up, and KW/BW were obviously decreased in rats of the CRS group (CRS + PAA group) after treating with PAA (Figures 2(a)–2(d)). In conclusion, the kidneys of CRS rats were obviously damaged and PAA treatment could significantly alleviate the renal damage in CRS rats.

The article "Poricoic Acid A Inhibits the NF-κB/MAPK Pathway to Alleviate Renal Fibrosis in Rats with Cardiorenal Syndrome" was retracted in 2023. Reasons: signs of a paper mill; suspected computer-generated content; unreliable results or conclusions; concerns about the data.

### 3.3. PAA Improves Renal Histopathological Damage and Renal Fibrosis in Rats with Cardiorenal Syndrome

To further observe the effect of PAA treatment on renal tissue damage in CRS rats, HE staining was performed on the renal tissue of each group of rats. The results displayed the normal morphology of glomeruli, renal tubules, and renal interstitium on the pathological sections of the rat kidneys in the Sham group and PAA group. However, renal tubular epithelial damage was observed in the renal tissue of the CRS group. Besides, renal tubules were significantly expanded, sclerotic, necrotic, tube formation occurred, and the interstitium was infiltrated by a large number of inflammatory cells. Nevertheless, compared with the CRS group, the damage of the renal tissue of the rats in the CRS + PAA group was obviously relieved and the renal tubule dilation and inflammatory cell infiltration were also improved (Figure 3(a)).

Masson staining was adopted to evaluate the degree of renal fibrosis in the rats in each group. The results showed the normal structure distribution and a small amount of collagen deposition for the renal tissue of rats in the Sham group and the PAA group. However, a large amount of collagen deposition was observed in the renal tissue of the CRS group, with severe fibrosis in glomeruli, renal tubules, and renal interstitium. Additionally, compared with the CRS group, the renal tissue of the CRS + PAA group exhibited obviously reduced collagen deposition and fibrosis (Figure 3(b)). We also measured the level of fibrosis-related proteins, *α*-SMA, and fibronectin in the kidney tissue of rats in each group. The results displayed that the expression level of *α*-SMA and fibronectin in the kidney tissue of the CRS group was significantly higher than that in the Sham group and the PAA group. Compared with the CRS group, the kidney tissue of CRS rats in the CRS + PAA group presented a significant reduction in the expression level of *α*-SMA and fibronectin (Figure 3(c)/3(d)). From the above analysis, PAA could not only effectively alleviate the pathological damage of renal tissue in CRS rats but also significantly improve renal fibrosis in CRS rats.

The article "Poricoic Acid A Inhibits the NF-κB/MAPK Pathway to Alleviate Renal Fibrosis in Rats with Cardiorenal Syndrome" was retracted in 2023. Reasons: signs of a paper mill; suspected computer-generated content; unreliable results or conclusions; concerns about the data.

### 3.4. PAA Inhibits the Inflammatory Response of Renal Tissue in Rats with Cardiorenal Syndrome

Studies reported the important role of the inflammatory response in organ damage in CRS [20]. To clear whether PAA could alleviate tissue damage by inhibiting inflammatory response, ELISA was utilized to detect the level of inflammatory factors (IL-1*β*, IL-6, and IL-10) in the kidney tissue of rats in each group. The results revealed that the level of IL-1*β* and IL-6 in renal tissue of the CRS group was a lot higher than that in the Sham group, while the level of IL-10 was obviously decreased (*P* < 0.01). Moreover, PAA treatment could notably reduce the level of IL-1*β* and IL-6 in the renal tissue of CRS rats and remarkably increase the level of IL-10 (*P* < 0.01) at the same time. Briefly speaking, PAA treatment could significantly inhibit the excessive inflammatory response in the kidneys of CRS rats (Figures 4(a)–4(c)).

### 3.5. PAA Inhibits NF-Κb/MAPK Signaling Pathway in Rats with Cardiorenal Syndrome

Studies stated the important role of NF-*κ*B and MAPK pathways in the inflammatory response of various diseases [21, 22]. However, the association between PAA relieving organ damage due to CRS by inhibiting inflammatory response and NF-*κ*B as well as the MAPK pathway still remained unclear. Therefore, the expression level of NF-*κ*B and MAPK signaling pathway-related proteins in the renal tissue of rats in each group was detected to further clarify the relation between PAA and pathways of NF-*κ*B and MAPK. The results displayed notably increased expression level of p-NF-*κ*B, p-IKB*α*, p-P38, and p-ERK and higher ratios of p-NF-*κ*B/NF-*κ*B, p-IKB*α*/IKB*α*, p-P38/P38, and p-ERK/ERK in the renal tissue of CRS rats compared with those of the Sham group (*P* < 0.01). While compared with the CRS group, the renal tissue of the CRS + PAA group presented obviously decreased the phosphorylation level of NF-*κ*B, IKB*α*, P38, and ERK (*P* < 0.01) and declined ratios of p-NF-*κ*B/NF-*κ*B, p-IKB*α*/IKB*α*, p-P38/P38, and p-ERK/ERK (Figures 5(a)–5(c)). From the above analysis, the NF-*κ*B/MAPK signaling pathway was remarkably activated in the renal tissue of CRS model rats and PAA treatment could significantly inhibit the activity of the NF-*κ*B/MAPK signaling pathway in the renal tissue of CRS rats.

## 4. Discussion

Natural products, applied in clinical practice for a long time, are considered as alternative therapies for the prevention and treatment of various kidney diseases [23]. Accumulating evidence suggests that many small-molecule compounds derived from natural products exert antifibrotic functions. Specifically, the antifibrotic functions of small-molecule compounds were achieved by improving the renin-angiotensin system, oxidative stress and inflammation, TGF-*β*/Smad and Wnt/*β*-catenin signaling pathway dysregulation, uremic toxin, amino acid, and lipid metabolism disorders [24]. Li et al. found that PAA protected H9c2 cardiomyocytes from lipopolysaccharide-induced cellular inflammatory response damage and inhibited cardiomyocyte apoptosis through inhibiting Erk1/2 and p38 pathways [25]. The above outcomes disclosed that PAA had a certain protective effect on the heart and kidney. This study also reported that PAA improved cardiac function in CRS rats and significantly increased LVEF and LVEDV, while decreased LVESV and LVPED. Besides, PAA could also improve renal pathological damage and relieve renal fibrosis. As a complex dynamic process, the formation and progression of renal fibrosis involves inflammatory cell infiltration, fibroblast activation and proliferation, ECM accumulation, tubular atrophy, and microvascular degeneration [26]. Also, dysregulation of inflammatory factors is one of the leading causes of renal fibrosis. Studies have revealed that the upregulation of IL-1*β* and IL-6 levels and the downregulation of IL-10 level are risk factors for renal fibrosis [27]. This study disclosed that PAA could exert anti-inflammatory effects by remarkably reducing the level of IL-1*β* and IL-6 in renal tissue and increasing the level of IL-10. The conclusion of this study is in line with the fact that PAA has beneficial effects on modulating inflammatory response in the body in many other research studies [28]. From the above outcomes, it can be speculated that PAA not only has a protective effect on heart and kidney damage in CRS but also can avoid further damage caused by inflammatory factors.

The article "Poricoic Acid A Inhibits the NF-κB/MAPK Pathway to Alleviate Renal Fibrosis in Rats with Cardiorenal Syndrome" was retracted in 2023. Reasons: signs of a paper mill; suspected computer-generated content; unreliable results or conclusions; concerns about the data.

NF-*κ*B is considered to be a typical proinflammatory signaling pathway. On the one hand, NF-*κ*B is mainly based on the activation of proinflammatory cytokines such as interleukin-1 (IL-1) and tumor necrosis factor alpha (TNF-*α*). On the other hand, NF-*κ*B can also promote the expressions of other proinflammatory genes, including cytokines, chemokines, and adhesion molecules [29]. Previous studies have revealed the important role of NF-*κ*B signaling pathway in heart and kidney-related diseases. For example, Deng et al. presented that higenamine may target the ASK1/MAPK (ERK and P38)/NF-*κ*B signaling pathway to improve cardiorenal function and alleviate cardiac and renal fibrosis in CRS rats. In addition, higenamine was also found to significantly inhibit the protein expression of mitogen-activated protein kinase (MAPK) (ERK and P38)/NF-*κ*B pathway in CRS rats and then to protect rat cardiomyocytes [30]. Cai et al. discovered that melatonin and exendin-4 treatment exerted protective effects on the heart of CRS rats through the TNF-*α*/NF-*κ*B/MMP-2/MMP-9/IL-1*β* pathway [31]. This study also showed that PAA inhibited the NF-*κ*B/MAPK signaling pathway in the renal tissue of CRS rats, thereby exerting a protective effect on the rat heart and kidney. Therefore, we speculated that the activation of NF-*κ*B/MAPK signaling pathway in CRS rats induced inflammatory response, thereby resulting in renal fibrosis and cardiorenal injury, while PAA could delay renal fibrosis and improve cardiorenal injury by inhibiting the NF-*κ*B/MAPK signaling pathway.

Chen et al. reported that the inhibition effect of PAA on renal fibrosis has concentration dependence [14]. Nevertheless, relevant exploration based on the concentration dependence was not performed in our study. Therefore, more detailed studies on dosage-efficacy relationship are needed. Furthermore, this study failed to verify that the PAA exerted anti-inflammatory and protective effects on heart and kidney injury through the NF-*κ*B/MAPK signaling pathway. Thus, it is necessary to evaluate the role of PAA after inhibition or activation of the pathway in CRS. Also, the specific interaction between PAA and NF-*κ*B/MAPK signaling pathway required further investigation. Additionally, as a formulated drug, “*Poria cocos* polysaccharide oral solution” was approved by the China Food and Drug Administration in 2015 for the treatment of various types of cancer, hepatitis, and other diseases, and “*Poria cocos* polysaccharide oral solution” can be applied alone or during chemoradiation for the treatment of cancer [11, 32]. Further improvement of the above experiments will be expected to provide strong support for PAA in the treatment of CRS.

## 5. Conclusion

To sum up, PAA can inhibit the level of IL-1*β* and IL-6 in the renal tissue of CRS rats and increase the level of IL-10, thereby inhibiting the renal inflammatory response. Moreover, PAA can also alleviate the pathological damage and fibrosis of the kidney and maintain heart and kidney function. The above functions of PAA may be related to the inhibitory effect on the NF-*κ*B/MAPK signaling pathway activity. In a word, PAA has the potential to serve as a CRS therapeutic drug.

## Figures and Tables

**Figure 1:** Poricoic acid A (PAA) improves cardiac function damage in rats with cardiorenal syndrome. (a-d) echocardiography to evaluate the changes of cardiac function indexes (LVEF, LVEDV, LVESV, and LVPED) of rats in each group; (e,f) HW/BW and LV/TL were calculated to evaluate the degree of cardiac hypertrophy and left ventricular hypertrophy in rats in each group. ^*∗∗*^*P* < 0.01*vs*. the Sham group; ^#^*P* < 0.05 and ^##^*P* < 0.01*vs*. the CRS group.

The article "Poricoic Acid A Inhibits the NF-κB/MAPK Pathway to Alleviate Renal Fibrosis in Rats with Cardiorenal Syndrome" was retracted in 2023. Reasons: signs of a paper mill; suspected computer-generated content; unreliable results or conclusions; concerns about the data.

**Figure 2:** Poricoic acid A (PAA) alleviates renal function damage in rats with cardiorenal syndrome. (a-c) biochemical test was applied to detect the level of renal function-related indexes (serum BUN, SCr, and urine 24-up) of rats in each group; (d) based on the measured kidney weight and the rat body weight, KW/BW was calculated to evaluate renal damage. ^*∗∗*^*P* < 0.01*vs*. the Sham group; ^##^*P* < 0.01*vs*. the CRS group.

**Figure 3:** Poricoic acid A (PAA) improves renal histopathological damage and renal fibrosis in rats with cardiorenal syndrome. (a) HE staining was adopted for evaluating the degree of tissue damage in the kidneys of rats in each group (200 ×); (b) Masson staining for the degree of fibrosis in the kidney tissue of rats in each group (200 ×); (c,d) Western blot for the protein expression level of *α*-SMA and fibronectin in kidney of rats in each group. ^*∗∗*^*P* < 0.01 vs. the Sham group; ^##^*P* < 0.01 vs. the CRS group.

**Figure 4:** Poricoic acid A (PAA) inhibits the inflammatory response in the renal tissue of rats with cardiorenal syndrome. (a-c) ELISA was applied to check the level of inflammatory factors in the renal tissue of rats in each group, including the level of proinflammatory factors (IL-1*β* and IL-6) and anti-inflammatory factor IL-10. ^*∗∗*^*P* < 0.01*vs*. the Sham group; ^##^*P* < 0.01*vs*. the CRS group.

**Figure 5:** Poricoic acid A (PAA) inhibits the NF-*κ*B/MAPK signaling pathway in renal tissue of rats with cardiorenal syndrome. (a-c) western blot was performed to detect the expression level of NF-*κ*B/MAPK signaling pathway-related proteins (p-NF-*κ*B, NF-*κ*B, p-IKB*α*, IKB*α*, p-P38, P38, p-ERK, and ERK) in renal tissue of rats in each group. ^*∗∗*^*P* < 0.01*vs*. the Sham group; ^#^*P* < 0.05*vs*. the CRS group.

## Data Availability

The data used to support the findings of this study are available from the corresponding author upon request.
